The article "CDCA4 suppresses epithelial–mesenchymal transtion (EMT) and metastasis in Non-small cell lung cancer through modulating autophagy" was published in 2021. Journal: Cancer Cell Int.

# CDCA4 suppresses epithelial–mesenchymal transtion (EMT) and metastasis in Non-small cell lung cancer through modulating autophagy

**DOI:** 10.1186/s12935-021-01754-w

**Published:** 2021-01-12

**Authors:** Chenxin Xu, Haixia Cao, Ying Sui, Hui Zhang, Chen Shi, Jianzhong Wu, Rong Ma, Jifeng Feng

**Affiliations:** 1 The Affiliated Cancer Hospital of Nanjing Medical University, Jiangsu Cancer Hospital & Jiangsu Institute of Cancer Research, No.42, Baiziting Street, Nanjing, 210009 Jiangsu China; 2 Research Center for Clinical Oncology, Jiangsu Cancer Hospital & Jiangsu Institute of Cancer Research & The Affiliated Cancer Hospital of Nanjing Medical University, Nanjing, 210009 Jiangsu China

**Keywords:** Non-small cell lung cancer, CDCA4, Migration and invasion, EMT, Autophagy, CARM1

## Abstract

**Background:**

Cell division cycle associated 4 (CDCA4) has been reported to be engaged into the progression of several cancers. The function of CDCA4 in Non-small cell lung cancer (NSCLC) was unknown. We aimed to explore the critical role of CDCA4 in NSCLC.

**Methods:**

CDCA4 stably knocking down and overexpression cell lines were established and Western blotting assay was applied to measure relevant protein expression of Epithelial-Mesenchymal Transtion (EMT) and cell autophagy. Staining of acidic vacuoles, transmission electron microscopy and immunofluorescence staining were employed to detect autophagy. The ability of cells to migrate and invade were detected by Transwell migration and invasion assays. The interaction of CDCA4 with CARM1 was identified by immunoprecipitation and Western blotting analysis.

**Results:**

In the present study, it was found that inhibition of CDCA4 induced EMT, migration and invasion of NSCLC cells while inhibiting autophagy of NSCLC cells. Meanwhile, overexpression of CDCA4 in NSCLC cells showed the opposite function. More importantly, the inhibition of autophagy could promote the EMT, migration and invasion of NSCLC cells, which should be impaired via the activation of autophagy. In addition, CDCA4-inhibited EMT, migration and invasion could be partially aggravated by autophagy activator, rapamycin, and reversed by autophagy inhibitor, 3-MA. Correspondingly, the application of rapamycin or 3-MA to CDCA4 knockdown cells showed the opposite effects. Further investigation suggested that CDCA4 could interact with coactivator associated arginine methyltransferase 1 (CARM1). Autophagy was induced while cell migration and invasion were inhibited in CARM1 knockdown cells. CDCA4 could suppress the protein expression CARM1 and knocking down of CARM1 could alter cell autophagy, migratory and invasive abilities regulated by CDCA4.

The article "CDCA4 suppresses epithelial–mesenchymal transtion (EMT) and metastasis in Non-small cell lung cancer through modulating autophagy" was published in 2021. Journal: Cancer Cell Int.

**Conclusion:**

All data indicated that CDCA4 inhibited the EMT, migration and invasion of NSCLC via interacting with CARM1 to modulate autophagy.

## Background

Lung cancer is the most commonly diagnosed cancer with the highest mortality among all cancers worldwide [1]. Although diagnostic and therapeutical techniques have been developing in recent years, lung cancer is predicted as a major disease burden continually well through the first half of this century [2]. Non-small cell lung cancer (NSCLC) is the most common form of lung cancer [3]. As cancer recurrence and metastasis are common incidents for patients with late stage of NSCLC, an improved understanding of the molecular mechanisms underlying NSCLC metastasis is of great significance to propose better therapeutic strategies, which are urgently required for prolonging patients overall survival.

Cell division cycle associated (CDCA) gene family serve as important regulators in many biological process, such as cell cycle [4]. Previous studies had indicated that some members of this gene family might have potential diagnostic and porgnostic values for both ovarian cancer [5] and hepatocellular carcinoma [6]. CDCA4, also known as HEPP/SEI-3/TRIP-Br3, is a member of CDCA gene family. Recently, several studies have shown that CDCA4 played various roles in different cancer types. In breast cancer CDCA4 could enhance cancer cell proliferation and reduce apoptosis [7]. Its role as cancer promoter was also reported in hepatocellular carcinoma [8]. However, CDCA4 worked as a tumor suppressor gene in cervical cancer as the knockdown of CDCA4 could promote cell proliferation [9]. The role of CDCA4 in NSCLC has not been well explored. Our study aims at filling in the gap in understanding the contribution of CDCA4 to NSCLC progression, which may provide basic molecular target for developing new therapeutic strategies for NSCLC.

Tumor metastasis is the leading cause of cancer deaths and regarded as an exacerbation of cancer progression. In the early stage of metastasis, cancer cells progress through the epithelial-to-mesenchymal transition (EMT), a process during which epithelial cells obtain semblable properties of mesenchymal cells with altered adhesive properties and motility [10] and thereby achieve increased migratory probability to invade surrounding tissues [11]. Autophagy is a conservative catabolic process wherein dysfunctional or damaged organelles and proteins are metabolically degraded as to maintain macromolecule synthesis [12]. Previous studies have demonstrated that autophagy functioned in cancer progression as a double-edged sword, as it may inhibit tumors in the development of cancers but enables tumor cell survival in stress [13]. Recently several researches indicate that autophagy is intricately involved in tumor metastasis, both with a EMT-promoting or EMT- restraining function [14–16]. However, the role and mechanism of CDCA4 in regulating autophagy during NSCLC metastasis are completely unclear.

The article "CDCA4 suppresses epithelial–mesenchymal transtion (EMT) and metastasis in Non-small cell lung cancer through modulating autophagy" was published in 2021. Journal: Cancer Cell Int.

In this study, we examined the functional relevance of CDCA4-associated autophagy in NSCLC, with a focus on EMT, tumor migration and invasion. Our results revealed that overexpression of CDCA4 could interact with coactivator associated arginine methyltransferase 1 (CARM1) and suppress its expression in NSCLC cells to induce autophagy, and as a result interfere with EMT and metastatic progression. Our data demonstrate for the first time that CDCA4-induced autophagy inhibits tumor cell migration and invasion in NSCLC, suggesting that CDCA4 may be a potential therapeutic target for NSCLC.

## Materials and methods

### Cell culture

Human Non-small cell lung cancer cell lines A549 and H1299 were obtained from Shanghai Cell Bank of the Chinese Academy of Sciences and cultured in RPMI-1640 medium with 10% fetal bovine serum (FBS; WISENT, Inc.). The cells were maintained in an environment of 5% CO_2_ at 37℃. Based on this culture environment, the medium of the cells was changed every three days.

### Quantitative PCR

Total RNA from cells was extracted using Takara MiniBEST Universal RNA Extraction Kit (Takara Biotechnology CO., Ltd) according to the manufacturer’s protocol. All PCR primers were designed and synthesized by Sangon Biotechnology Co. (Shanghai, China), according to the gene sequences in Genbank. After the concentration and quality of RNA was determined by 260/280 nm absorbance, PrimeScript RT Master mix (Takara Biotechnology CO., Ltd) was applied to reverse transcribe RNA into high-capacity DNA. Quantitative PCR reaction was performed on an ABI 7300 PCR System (Applied Biosystems, CA, USA) using a SYBR Green Master Mix (Thermo Fisher Scientific, USA). Relative expression was normalized to β-Actin as an internal control and calculated using 2^−△△^ CT.

### Western Boltting analysis

Cells were lysed with ice-cold radio-immunoprecipitation assay (RIPA) buffer (Beyotime Biotechnology, Jiangsu, China) containing proteinase inhibitors. The cell lysate was scraped and centrifuged for 20 min, 12000*g* at 4 ℃. The supernatants were retained and concentrations were determined using a BCA protein assay kit (Beyotime Biotechnology, Jiangsu, China). Equal amounts of protein were loaded in SDS-PAGE gels and separated by electrophoresis. After electrophoresis, the proteins were transferred on a polyvinylidene fluoride (PVDF) membrane. Then the membranes were blocked at room temperature for 1 h with 5% BSA, and then incubated with anti-CDCA4 antibody (cat. no. 11625-1-AP; 1:1000; Proteintech, Inc.), anti-LC3B antibody (cat. no. 3865; 1:1000; Cells Signaling Technology, Inc.), anti-P62 (cat. no. 18420-1-AP; 1:1000; Proteintech, Inc.), anti-N-Cadherin (cat. no. 13116; 1:1000; Cells Signaling Technology, Inc.), anti-E-Cadherin (cat. no. 3195; 1:1000; Cells Signaling Technology, Inc.), anti-Snail (cat. no. 3879; 1:1000; Cells Signaling Technology, Inc.), anti-Vimentin (cat. no. 5741; 1:1000; Cells Signaling Technology, Inc.) and anti-β-Actin (cat. no. 20536–1-AP; 1:1000; Proteintech, Inc.) overnight at 4 ℃. After being washed in TBS-T, membranes were incubated with an HRP-conjugated secondary antibody for 1 h at room temperature. Then the membranes were visualized by chemiluminescent reagents (Millipore, USA).

The article "CDCA4 suppresses epithelial–mesenchymal transtion (EMT) and metastasis in Non-small cell lung cancer through modulating autophagy" was published in 2021. Journal: Cancer Cell Int.

### Trans-well assay

Certain number of 2 × 10^4^ cells/well were resuspended in 200 µl of serum-free medium in the upper chamber (8-µm pore size, Coster, Corning, USA) and the lower chamber was filled with 600 µl of medium supplemented with 10% FBS. After incubation for 24 h (migration assay) or 48 h (invasion assay) at 37℃, the cells in the parietal chamber were removed with a wet cotton swab and cells on the submucosal surface were immobilized in 4% paraformaldehyde for 30 min. Then the cells were stained with a crystal violet solution. The number of migrated cells was quantified under a microscope by counting those in four random fields of each membrane. Three independent experiments were performed.

### Lentiviral production and stable cell line construction

Lentiviral vectors expressing shRNA and CDCA4 were obtained from Vigene Biosciences China. A549 and H1299 cells were cultured overnight on 6-well plates then transduced by the above lentiviruses. After incubating for 24 h, cells were selected with 2 mg/ml puromycin for A549 cell and 4 mg/ml puromycin for H1299 cell for 3 days. Stable cell lines were harvested.

### Staining of acidic vacuoles

Cells were cultured overnight on 6-well flat cover slides, washed with PBS for three times then stained with 1 µM AO (Solarbio, Beijing China) for 15 min at 37 ℃. Then cells were washed with PBS for three times and observed with Axio scope A1.

### TEM (Transmission Electron Microscopy)

A549 cells were digested and then fixed with 2.5% glutaraldehyde overnight at 4℃. After washing the cells with PBS (0.1 mol/L) for 4 times (15mins/time), 1% osmium tetroxide was used to fix the cells for 2 h at 4℃ and acetone (50, 70, 90 and 100%) for 15 min each was used to dehydrate the cells. After dehydration, samples were permeated with 100% acetone and epoxy resin (1:1) for 2 h and then 100% acetone and epoxy resin (1:2) for 2 h, following by permeated with pure epoxy resin overnight then embedded in epoxy resin (Epon 812) and polymerized in drying oven (12 h at 37 ℃, 12 h at 45 ℃ and 48 h at 60 ℃). Ultra-thin sections (60 nm) were prepared using an ultramicrotome (Leica Ultracut R) and stained with uranyl acetate and lead nitrate. The images were captured at ×20,000 magnification on a Transmission Electron Microscope (JEM-1010, JEOL) installed in the Analysis and Testing Center in Nanjing Medical University.

The article "CDCA4 suppresses epithelial–mesenchymal transtion (EMT) and metastasis in Non-small cell lung cancer through modulating autophagy" was published in 2021. Journal: Cancer Cell Int.

### Immunofluorescence staining

Cells were cultured on glass coverslips overnight. After being washed with PBS for three times, 4% paraformaldehyde was added for 15 min to immobilize cells at room temperature. Then cells were washed three times with ice-cold PBS and incubated with 0.5% Triton X-100 in PBS at room temperature for 20 min. After incubation, cells were washed with PBS and then blocked with 3% bovine serum albumin for 30 min. Cells were incubated with anti-LC3B antibody (cat. no. 3865; 1:200; Cells Signaling Technology, Inc.) and anti-P62 (cat. no. 18420–1-AP; 1:200; Proteintech, Inc.) in 4℃ overnight. After being washed with PBS-T for three times, cells were incubated with Cy3 conjugated Goat Anti-Rabbit IgG (1:300; GB21303; Servicebio) and Cy5 conjugated Goat Anti-Rabbit IgG (1:500; GB27303; Servicebio) for 50 min at room temperature. 4′, 6-Diamidino-2-phenylindole (Servicebio Biotechnology) was added for 10 min. Images were captured using a fluorescence microscope (Nikon Eclipse C1; Nikon Corporation).

### Immunoprecipitation

An immunoprecipitation (IP) assay was performed using the Thermo Scientific™ Pierce Classic IP Kit (Thermo Fisher Scientific, MA, USA) accroding to the manufacturer’s instructions. A549 cells with CDCA4 overexpression were lysed in IP Lysis containing protease inhibitors and centrifuged for 15mins, 12000 g at 4℃. The supernatants were incubated with diluted anti-IgG antibody (cat. no. sc-2025; 5 µg; Santa Cruz Biotechnology, Inc.), anti-CDCA4 antibody (cat. no. 11625--AP; 5 µg; Proteintech, Inc.) and anti-CARM1 antibody (cat. no. 55246-1-AP; 5 µg; Proteintech, Inc.) and the magenetic beads overnight at 4 ℃. After washing, the proteins were eluted with 2× SDS-PAGE Sample Loading Buffer ( Beyotime Biotechnology, Jiangsu, China) for 10 min at 100 ℃. Immunocomplexes were analyzed by SDS/PAGE and immunoblotting with anti-CDCA4 and anti-CARM1 antibody.

### Statistical analysis

Statistical analyses were performed using GraphPad Prism version 6 statistical software.All data shown represent the results obtained from triplicate independent experiments with mean ± SD. Student’s *t*-test was used to evaluate comparisons between two groups. P < 0.05 was set to indicate a statistically significant difference.

The article "CDCA4 suppresses epithelial–mesenchymal transtion (EMT) and metastasis in Non-small cell lung cancer through modulating autophagy" was published in 2021. Journal: Cancer Cell Int.

## Results

### CDCA4 suppresses EMT, migration and invasion in NSCLC cells

According to the relative expression quantity of CDCA4 on both mRNA and protein level (Fig. 1a, b), H1299 and A549 cell lines were selected to perform subsequent experiments as the abundance of CDCA4 was high in H1299 and medium in A549. We next establish CDCA4 stably knockdown H1299 cell line and CDCA4 stably overexpression A549 cell line. Western blotting and q-PCR confirmed the successful modulation of CDCA4 expression level in these cells (Fig. 1c, d). We then used these cells for in vitro analysis of NSCLC cell migration and invasion. Results showed that CDCA4 knockdown improved migrative and invasive abilities of H1299 cell, while CDCA4 overexpression impaired migration and invasion of A549 cell (Fig. 2a). As the phenomenon of epithelial-mesenchymal transition (EMT) commonly occur during tumor metastasis, we measured the expression pattern of classic EMT markers. Western blot assay results showed that in the shCDCA4 cells epithelial markers such as E-cadherin decreased while mesenchymal markers such as N-cadherin, Vimentin and Snail increased. The results were coincident in CDCA4-overexpressing cell lines, as the expression level of above EMT markers were reversed correspondingly (Fig. 2b). Collectively, these findings suggested that CDCA4 was a blocker of NSCLC EMT, migration and invasion.

**Fig. 1:** Stable cell line was established. **a** Quantitative PCR (qPCR) analysis of CDCA4 basal mRNA expression in six NSCLC cell lines. CDCA4 mRNA expression levels were normalized according to the β-actin expression level. **b** Western blotting analysis of CDCA4 basal protein expression in the six cell lines; β-actin was used as a loading control. **c** qPCR analysis and western blotting analysis of efficiency of knocking down CDCA4 in H1299 cells. **d** qPCR analysis and western blotting analysis of efficiency of overexpression of CDCA4 in A549 cells. Data are means ± S.D. ***P < 0.005

**Fig. 2:** CDCA4 inhibits the EMT, migration and invasion of NSCLC. **a** Comparison of the migration and invasion of H1299 and A549 cells using transwell compartments. **b** Western blotting analysis of E-cad, N-cad, Vimentin and Snail protein expression. β-actin was used as a loading control. Data are means ± S.D. *P < 0.05, **P < 0.01, ***P < 0.005

### CDCA4 expression levels affect NSCLC autophagy

The association between tumor autophagy and tumor metastasis has been explored in many studies recently. As CDCA4 has previously been shown to serve as an autophagy regulator, we propose a hypothesis that autophagy played a crucial role in the process of CDCA4 regulating EMT, migration and invasion of NSCLC cells. Compared with cells transfected with vector, the formation of autophagosomes was increased in CDCA4 overexpressing A549 cells stained with acridine orange, as more amounts of acidic vacuoles could be counted in sight. In CDCA4 knockdown H1299 cells the formation of autophagosomes showed the opposite change (Fig. 3a). TEM showed the consistent phenomenon of activation of autophagic flux with accumulation of autophagic vacuoles containing intracellular material in CDCA4 overexpressing A549 cells (Fig. 3b). Moreover, an elevated immunofluorescence signal of LC3B and a weakened signal of P62 were observed in CDCA4 overexpressing A549 cell line compared with vector. The changes were correspondingly reversed in CDCA4 inhibition H1299 cells (Fig. 3c). As presented in Fig. 3d, western blotting assay showed that the expression of LC3B decreased and P62 showed the opposite change with the knocking down of CDCA4, along with other autophagy-associated markers such as BECLIN-1, ATG5 and ATG7 decreased. CDCA4 overexpressing cells showed consistent changes in protein levels of above markers. Overall, these results confirmed that CDCA4 positively modulated the autophagy pathway in NSCLC cells.

The article "CDCA4 suppresses epithelial–mesenchymal transtion (EMT) and metastasis in Non-small cell lung cancer through modulating autophagy" was published in 2021. Journal: Cancer Cell Int.

**Fig. 3:** CDCA4 induces autophagy in NSCLC cells. **a** The effect of CDCA4 on the formation of acidic vacuoles was shown. Yellow to orange dots in the cytoplasm represented acidic vacuoles. Representative images were shown. **b** Electron microscopy showed the different autophagic activation in A549 CDCA4 overexpression cells. **c** Immunocytochemistry assay detected an elevated signal of LC3B and reduced signal of P62 in A549 CDCA4 overexpression cell. In H1299 CDCA4 knocking down cell a reduced signal of LC3B and elevated signal of LC3B were detected. **d** Western blotting analysis of P62, LC3B, Beclin-1, ATG5 and ATG7 protein expression. β-actin was used as a loading control. Data are means ± S.D. **P < 0.01, ***P < 0.005

### Autophagy modulates EMT of NSCLC cells

In order to explore the role of autophagy in EMT, A549 and H1299 NSCLC cells were treated with rapamycin or 3-MA, respectively known as autophagy activator and inhibitor, in indicated concentration for 48 h. The expression levels of LC3B increased markedly while P62 protein expression significantly decreased after cells treated with rapamycin (Fig. 4a). With the treatment of 3-MA for 48 h, the expression pattern of both A549 and H1299 reversed (Fig. 4c), indicating that rapamycin could stimulate cell autophagy while 3-MA could suppress cell autophagy in NSCLC cells. As shown in Fig. 4a, c, expression of EMT markers altered in cells treated with rapamycin or 3-MA. In addition, Trans-well assay indicated that activation of autophagy blocked cell migration and invasion while inhibition of autophagy had the opposite effect (Fig. 4b, d). The overall results suggested that autophagy could act as a regulator of NSCLC EMT.

The article "CDCA4 suppresses epithelial–mesenchymal transtion (EMT) and metastasis in Non-small cell lung cancer through modulating autophagy" was published in 2021. Journal: Cancer Cell Int.

**Fig. 4:** Activation or inhibition of autophagy alters the EMT, migration and invasion of NSCLC cells. A549 and H1299 cells were treated with dimethyl sulfoxide (control) or rapamycin (100 nM) for 48 h. **a** Western blotting analysis of P62, LC3B, E-cad, N-cad and Snail protein expression. β-actin was used as a loading control. **b** Comparison of the migration and invasion of A549 and H1299 cells using transwell compartments. A549 and H1299 cells were treated with phosphate-buffered saline (control) or 3-methyladenine (5 mM) for 48 h. **c** Western blotting analysis of P62, LC3B, E-cad, N-cad and Snail protein expression. β-actin was used as a loading control. **d** Comparison of the migration and invasion of A549 and H1299 cells using transwell compartments. Data are means ± S.D. *P < 0.05, **P < 0.01, ***P < 0.005

### Effects of autophagy activation on CDCA4-modulated EMT, migration and invasion in NSCLC cells

To investigate whether autophagy is the pathway through which CDCA4 restained EMT and consequently blocked the migration and invasion of NSCLC cells, we treated CDCA4 overexpressing A549 cells or CDCA4 knockdown H1299 cells with autophagy agnosit respectively. As the primary target of rapamycin (mTOR) is regarted as a key regulator of autophagy, We chose to use rapamycin treatment with the aim of inducing autophagy in treated cells. It was observed that with the treatment of rapamycin, the increased LC3B protein expression while decreased P62 protein expression induced by CDCA4 overexpression were aggravated in A549 cells (Fig. 5a). Moreover, the weakened ability of migration and invasion in CDCA4 overexpressing A549 cells was further diminished by application of rapamycin (Fig. 5b). Western blotting assay showed decreased expression of N-cadherin as well as dramatically downregulated Snail expression, while increased expression of E-cadherin (Fig. 5a). In CDCA4 knocking down cells, the treatment of rapamycin showed a reversed effect on decreased LC3B protein expression and increased P62 protein expression (Fig. 5c). Together with Trans-well assay verified that the shCDCA4-improving abilities of migration and invasion were weakened in H1299 cells (Fig. 5d). Meanwhile, more significant gap in protein expression differences of EMT markers also assisted in verifying that rapamycin could partly reverse CDCA4 knockdown-promoted EMT, migration and invasion in H1299 cells (Fig. 5c). Taken together, our results demonstrated that EMT, migration and invasion inhibited by CDCA4 could be aggraveted by arousing autophagy in NSCLC, while downregulation of CDCA4 promoted.migration could be blocked via autophagy activation.

The article "CDCA4 suppresses epithelial–mesenchymal transtion (EMT) and metastasis in Non-small cell lung cancer through modulating autophagy" was published in 2021. Journal: Cancer Cell Int.

**Fig. 5:** Effects of CDCA4 on EMT, migration and invasion could be influenced by autophagy activation. CDCA4 overexpressing and control A549 cells were treated with dimethyl sulfoxide (control) or rapamycin (100 nM) for 48 h. **a** Western blotting analysis was used to assess the expression of the indicated proteins in treated A549 cells. β-actin was used as a loading control. **b** Cell migration and invasion assays were performed using transwell compartments. CDCA4 knocking down and control H1299 cells were treated with dimethyl sulfoxide (control) or rapamycin (100 nM) for 48 h. **c** Western blotting analysis was used to assess the expression of the indicated proteins in treated H1299 cells. β-actin was used as a loading control. **d** Cell migration and invasion assays were performed using transwell compartments. Data are means ± S.D. *P < 0.05, **P < 0.01, ***P < 0.005

### The inhibition of autophagy reverses CDCA4-suppressed EMT, migration and invasion in NSCLC cells

As we have proved that activation of autophagy had an influence on CDCA4-regulated EMT, migration and invasion in NSCLC, the flipside of autophagy was also investigated using 3-methyladenine (3-MA), which is a class III phosphatidylinositol 3-kinase (Ptdlns3K) inhibitor, to treat both A549 and H1299 cells. In A549 cells, the CDCA4 overexpression-midiated anti- metastasis effects were reversed when cells were treated with the autophagy inhibitor 3-MA (Fig. 6b). In addition, changes in protein expression of assocaited EMT markers were exhibited in Fig. 6a. In H1299 cells co-treated with shCDCA4 and 3-MA, western blotting assay showed further downregulation of LC3B expression and upregulation of P62 expression (Fig. 6c). Enhanced cell migration and invasion were observed in CDCA4 knocking down cells but not control cells (Fig. 6d), together with significantly increased protein expression of markers of mesenchymal cells ( N-cadherin and Snail) and decreased expression of E-cadherin, which marks epithelial cells (Fig. 6c). These data indicated that CDCA4-suppressed EMT, migration and invasion in A549 and H1299 cells could be reversed by the inhibition of autophagy. Collectively, our results suggested that the inhibitory effects of CDCA4 on the migration and invasion abilities of NSCLC cells likely worked through the autophagy-EMT pathway.

The article "CDCA4 suppresses epithelial–mesenchymal transtion (EMT) and metastasis in Non-small cell lung cancer through modulating autophagy" was published in 2021. Journal: Cancer Cell Int.

**Fig. 6:** Effects of CDCA4 on EMT, migration and invasion could be affected by autophagy inhibition. CDCA4 overexpressing and control A549 cells were treated with phosphate-buffered saline (control) or 3-methyladenine (5 mM) for 48 h. **a** Western blotting analysis was used to assess the expression of the indicated proteins in treated A549 cells. β-actin was used as a loading control. **b** Cell migration and invasion assays were performed using transwell compartments. c,d. CDCA4 knocking down and control H1299 cells were treated with phosphate-buffered saline (control) or 3-methyladenine (5 mM) for 48 h. **c** Western blotting analysis was used to assess the expression of the indicated proteins in treated H1299 cells. β-actin was used as a loading control. **d** Cell migration and invasion assays were performed using transwell compartments. Data are means ± S.D. *P < 0.05, **P < 0.01, ***P < 0.005

### CDCA4 interacts with CARM1 and suppresses CARM1 protein expression

We next explored the underlying molecular mechanism of CDCA4 inducing autophagy through performing IP assay with CDCA4 overexpressing A549 cells and subjected the binding proteins to mass spectrometry. After literature search of regulatory roles in autophagy and CO-IP assay to verify the combinational relation with CDCA4, we confirmed that CARM1 as a binding partner of CDCA4 (Fig. 7a) and there was possibility that CDCA4 could regulate autophagy through interacting with CARM1. Western blotting assay showed that CDCA4 could negatively regulate the protein expression of CARM1 (Fig. 7b) and after knocking down CARM1 with siRNA, the decreased expression of P62 and increased expression of LC3B were shown in both A549 and H1299 cell lines (Fig. 7c, d). These data indicated that CARM1 served as a suppressor of autophagy in NSCLC cells, suggesting that CDCA4 may induce autophagy through suppressing the protein expression of CARM1. With the inhibition of migration and invasion in CARM1 knocking down cells (Fig. 7e), we proposed a hypothesis that CDCA4 could suppress NSCLC migration and invasion through downregulating CARM1 to promote autophagy.

**Fig. 7:** CDCA4 interacts with CARM1 and suppresses CARM1 expression. **a** CO-IP assays were performed in A549 CDCA4 overexpressing cells. **b** Western blotting. analysis was used to assess the expression of CARM1 and CDCA4 in CDCA4 overexpressing cells or knocking down cells. β-actin was used as a loading control. **c** Western blotting analysis and qPCR analysis of efficiency of knocking down CDCA4 in both A549 and H1299 cells. **d** Western blotting analysis of P62 and LC3B protein expression. β-actin was used as a loading control. **e** Cell migration and invasion assays were performed using transwell compartments. Data are means ± S.D. *P < 0.05, **P < 0.01, ***P < 0.005

The article "CDCA4 suppresses epithelial–mesenchymal transtion (EMT) and metastasis in Non-small cell lung cancer through modulating autophagy" was published in 2021. Journal: Cancer Cell Int.

### CARM1 impacts the ability of CDCA4 to control NSCLC migration, invasion and autophagy

To explore if CARM1 was the downstream functional molecule through which CDCA4 could control NSCLC migration, invasion and autophagy, we performed rescue assay via knocking down CARM1 with specific siRNA in both CDCA4 overexpressing cells and CDCA4 knocking down cells to see alterations in migration and autophagy. Results showed that in CDCA4 overexpressing cells, CARM1 knocking down further increased LC3B expression as well as decreased P62 expression (Fig. 8a). Together with autophagy promotion was the more evidently inhibition of migration and invasion (Fig. 8b). Meanwhile, the downregulation of CARM1 could reverse both the inhibition of autophagy or the promotion of NSCLC migration and invasion caused by CDCA4 knocking down (Fig. 8c, d). These data demonstrated that CARM1 could impact the ability of CDCA4 to induce autophagy and suppress migration or invasion in NSCLC, suggesting that CARM1 may serves as the downstream functional molecule of CDCA4. CARM1 has been reported exerting a transcriptional co-activator function on autophagy-related genes under glucose starvation condition. However in this study, we found that with CARM1 knocking down the alterations in mRNA level of a few common autophagy-associated genes showed no consistency in both A549 and H1299 cell lines (Fig. 8e). This suggested that CARM1 may not served as a transcriptional regulator in NSCLC cells under nutritional sufficient conditions. The underlying mechanism of CARM1 regulating autophagy requires further investigation.

**Fig. 8:** CARM1 knockdown could alter the functions of CDCA4 both in inducing autophagy and suppressing migration. b. CDCA4 overexpressing and control A549 cells were transfected with siCARM1. **a** Western blotting analysis was used to assess the expression of the indicated proteins in treated A549 cells. β-actin was used as a loading control. **b** Cell migration and invasion assays were performed using transwell compartments. c.d. CDCA4 knocking down and control H1299 cells were transfected with siCARM1. **c** Western blotting analysis was used to assess the expression of the indicated proteins in treated A549 cells. β-actin was used as a loading control. **d** Cell migration and invasion assays were performed using transwell compartments. **e** qPCR analysis of seven autophagy-related genes. Data are means ± S.D. *P < 0.05, **P < 0.01, ***P < 0.005

## Discussion

Cell division is a process during which large numbers of cells are produced for organism living. However, abnormal cell division can contribute to a variety of cancer-promoting errors. The accumulation of these errors could further promote cell division under permissive extracellular environments, and eventually trigger the formation and growth of abnormal cell populations that initiate tumorigenesis [17]. As a result, it is inferred that cell division associated proteins are of great significance in digging in underlying mechanisms of oncogenesis and development of malignant tumors. Cell division cycle associated protein 4 (CDCA4) has been proved as an potential tumor promoter in various cancer types. As an E2F transcription factor family-induced nuclear factor, CDCA4 could function in regulating E2F-dependent transcriptional activation and cell proliferation[9]. Besides, CDCA4 was characterized as a regulator of p53 transcriptional activity but regulates cell growth in a p53-independent way [18]. Although previous studies have demonstrated that CDCA4 could promote cell proliferation in human breast cancer and maligant melanoma, its other potential influence on tumor progression is still unclear. In addition, the potential effects of CDCA4-induced stimulation of transactivation function of p53 are also unexplored. Herein we specifically assessed the role of CDCA4 in NSCLC metastasis and investigated the underlying mechanism. We found that knockdown of CDCA4 enhanced its ability in promoting migration and invasion in an EMT-dependent manner through a mechanism at least partially dependent upon the inhibition of autophagy, with CDCA4 overexpression showing the opposite effect. Beyond that, our results demonstrated that CDCA4 had the ability of inhibiting metastasis in NSCLC cells in a p53-independent manner, as the two NSCLC cell lines we chose to carry out experiments were A549, which contain wild p53 type, and H1299, in which p53 is deficient, and results suggested that CDCA4 had the same function in inhibiting migration and invasion in both cell lines. Although p53 could regulate a few key stages of metastatic progression such as cell migration and invasion [19], distinct p53 expression status in these two cell lines showed little different effects on NSCLC metastasis, indicating that p53 pathway is not the key pathway through which CDCA4 functions as a cancer metastasis regulator. Our further data demonstrated that CDCA4 could inhibit cell migration and invasion via autophagy pathway. To our knowledge, this is the first report specifically report the function of CDCA4 in NSCLC metastasis and its regulatory role in regulating autophagy. In addition, this is the first report showing the relevance between CDCA4-inhibited migration and autophagy.

The article "CDCA4 suppresses epithelial–mesenchymal transtion (EMT) and metastasis in Non-small cell lung cancer through modulating autophagy" was published in 2021. Journal: Cancer Cell Int.

In previous studies, CDCA4 was proved as a tumor promoter in various cancers, representing as an attractive therapeutic target. Its role in promoting cancer cells proliferation in other cancer types have been studied extensively, little is known about the potential role of CDCA4 in cancer progression, especially in the metastasis of NSCLC. The purpose of this article is to explore the effects and underlying mechanisms of CDCA4 on the metastasis of NSCLC. After establishing CDCA4 stably knocking down or overexpression cell lines, we used Tran-swell assays to investigate the role of CDCA4 in migration and invasion. Our results showed that overexpression of CDCA4 could significantly impair NSCLC migration and invasion capability in vitro, whereas its downregulation could dramatically promote NSCLC migration and invasion in vitro. Accordingly these results identify a negatively-regulating role of CDCA4 in NSCLC metastasis. In recent years, increasing incidence of NSCLC implies the significance of identifying more accurate tumor biomarkers and improving current precise treatment strategies. Identification of key molecules of NSCLC metastasis can benefit not only in predicting the metastasis trend of primary tumor, according to which more specific excision extension in lung cancer resection as well as range of radiotherapy can be determined, but also in treating patients with targeted therapies when NSCLC recur with metastasis. Our studies have suggested that CDCA4 is associated with NSCLC migration and invasion in vitro, further studies in vivo should be done to prove CDCA4 as a potential biomarker of NSCLC metastasis.

EMT programmes have been pointed as integral components of the malignant progression of almost all types of carcinoma [20]. During this programme, cancer cells evolve the ability to migrate through the body cavity, with the morphological and functional transformation from epithelial cell to mesenchymal cell [21]. The properties of mesenchymal cell include reduced adhesion and enhanced motility, which allow cancer cells presenting an more aggressive and invasive phenotype [22]. Several molecular markers for EMT have been defined, such as increased expression of N-cadherin and Vimentin, increased production of the transcription factors like Snail and inhibited production of E-cadherin [23]. In this report, we found that overexpression of CDCA4 led to increased expression of E-cadherin and reduced N-cadherin, Vimentin and Snail expression in NSCLC cells, while downregulation of CDCA4 confers the opposite effects. This thus suggested that CDCA4 inhibited the EMT in NSCLC cells, highlight a highly potential link between CDCA4 and the metastasis of NSCLC.

The article "CDCA4 suppresses epithelial–mesenchymal transtion (EMT) and metastasis in Non-small cell lung cancer through modulating autophagy" was published in 2021. Journal: Cancer Cell Int.

Autophagy is a cellular spontaneous process during which intracellular proteins and organelles are captured and degraded as to sustain metabolism and homeostasis in the starved environment. In cancer, autophagy could be neutral, tumor-suppressive or tumor-promoting in different contexts [24]. Although in most contexts, autophagy facilitates tumorigenesis by supplying materials to cancer cells for their increased metabolic and biosynthetic demands imposed by deregulated proliferation, in some contexts autophagy also suppresses tumorigenesis as autophagy deficiency could cause oxidative stress, activation of the DNA damage response and genome instability, which are known cause of cancer initiation and progression [25]. Autophagy also play a critical role in regulating tumor cell migration and invasion, but the association between autophagy and EMT remains controversial. On the one hand, increasing evidence such as turnover of components of the cell migration machinery and EMT proteins has emerged to demonstrate that autophagy could promote tumor metastasis through inducing EMT [26], on the other hand autophagy modulation was reported with the effect of triggering a molecular switch from a mesenchymal phenotype to an epithelial-like one, consequently impaired migration and invasion in different contexts [27, 28]. As it has been reported that CDCA4 served as a regulator of cell apoptosis via autophagy pathway in various cancers [29], we supposed that the regulatory mechanism of CDCA4 on cell migration and invasion partly contained regulation of autophagy. Specifically, our data demonstrated that CDCA4 overexpression upregulated the protein expression of classical autophagy marker such as LC3B along with downregulation of P62. Together with these changes common markers of autophagy pathway such as Beclin-1, ATG5 and ATG7 also altered correspondingly. These results suggested that CDCA4 had the property of inducing autophagy. To further investigate whether autophagy had an effect on NSCLC cell migration and invasion, we respectively dealt cells with rapamycin as autophagy activator or 3-MA as autophagy inhibitor and then detect the migration capacity alteration of both cells. We found that in vitro, induction of autophagy resulting in inhibition of cell migration and invasion in NSCLC, and inhibition of autophagy showed the opposite results. Along with alterations in protein expression, our data demonstrated that autophagy regulation served as an EMT modulator in NSCLC cells. Further investigation was set on whether CDCA4 could inhibit cell migration and invasion through autophagy pathway. We found that inducing autophagy via overexpressing CDCA4 was linked to a partial EMT phenotypic reversion within NSCLC cells, which phenomenon can be strengthened by further activating autophagy, while impairing autophagy in these cells could reverse the observed defects in migration and invasion upon CDCA4 overexpression in vitro. Reducing autophagy via knocking down CDCA4 showed the opposite alteration of EMT markers in NSCLC cells, while 3-MA and CDCA4 knockdown synergistically enhanced the invasive effects of NSCLC cells. In addition, combination therapy significantly promoted EMT compared to treatment alone. As a result, we hypothesized that applying autophagy activators to CDCA4 high expression patients could reverse EMT and significantly prevent NSCLC cell invasion due to its enhanced anti-invasive effect.

The article "CDCA4 suppresses epithelial–mesenchymal transtion (EMT) and metastasis in Non-small cell lung cancer through modulating autophagy" was published in 2021. Journal: Cancer Cell Int.

CARM1 is known as a crucial component of autophagy in mammals with the transcriptional co-activator function on autophagy-related genes through transcription factor EB (TFEB) [30, 31]. Through mediating methylated modification of BAF155 and PKM2, CARM1 could enhance breast cancer progression and metastasis [32, 33]. In NSCLC, CARM1 also serves as a tumor promoter [34]. Here, we found that CDCA4 could interact with CARM1 and suppress the protein expression of CARM1. However, with CARM1 knocking down we found that autophagy was promoted in both A549 and H1299 cell lines, which is opposite to previous studies. This is a very interesting phenomenon and we inferred that it is because the condition in previous studies was glucose starvation but in our studies was nutritional sufficient condition. To verify CARM1 as a downstream functional molecule of CDCA4, we performed rescue assay and found CARM1 knockdown could alter effects on cell autophagy, migration and invasion caused by CDCA4. These results demonstrated that CDCA4 could induce autophagy through suppressing expression of CARM1, thus inhibiting NSCLC migration and invasion. Nevertheless, we also found that the knocking down of CARM1 did not alter mRNA expression of several common autophagy-related genes, which means that CARM1 may not serve as the transcriptional co-activator in NSCLC under our nutritional sufficient condition. The specific underlying mechanism of CARM1 inhibiting autophagy requires further investigation.

In conclusion, these results suggest a potential model whereby CDCA4 promotes NSCLC cell autophagy, thus inhibiting the migration and invasion of these cells. For future work, vivo experiments will be conducted to test whether the effect of CDCA4 on migration and invasion and its regulation of autophagy are consistent with the results of in vitro experiments. Overall, the present study not only suggests that CDCA4 could inhibit EMT, migration and invasion of NSCLC cells, but also provides a novel role for autophagy in these processes. In addition, the present study demonstrates the potential of identifying novel molecular targets, providing a basis for future investigations of more beneficial clinical strategies for NSCLC treatment.

The article "CDCA4 suppresses epithelial–mesenchymal transtion (EMT) and metastasis in Non-small cell lung cancer through modulating autophagy" was published in 2021. Journal: Cancer Cell Int.

## Conclusion

The findings of this study demonstrate that CDCA4 serves as a tumor suppressor in NSCLC, with the function of inhibiting migration and invasion of NSCLC through modulating the autophagy pathway. As inactivation of tumor suppresser genes is an important mechanism of tumorigenesis and progression, this study may provide valuable reference for early diagnosis, monitoring progression and evaluating prognosis of NSCLC.

## Data Availability

All data generated or analyzed during this study are included in this article.

## Abbreviations

CDCA4: Cell division cycle associated 4
CARM1: Coactivator associated arginine methyltransferase 1
EMT: Epithelial-to-mesenchymal transition
NSCLC: Non-small cell lung cancer
3-MA: 3-Methyladenine
Ptdlns3K: Phosphatidylinositol 3-kinase
TFEB: Transcription factor EB
